The article "Pulmonary artery sarcoma with angiosarcoma phenotype mimicking pleomorphic malignant fibrous histiocytoma: a case report" was published in 2012. Journal: Diagn Pathol.

# Pulmonary artery sarcoma with angiosarcoma phenotype mimicking pleomorphic malignant fibrous histiocytoma: a case report

**DOI:** 10.1186/1746-1596-7-154

**Published:** 2012-11-07

**Authors:** Olga L Bohn, Eric Acosta-Ponce de León, Oscar Lezama, Nina P Rios-Luna, Sergio Sánchez-Sosa, Antonio Llombart-Bosch

**Affiliations:** 1 Department of Pathology, Christus Mugerza UPAEP University Hospital, Puebla, 72000, Mexico; 2 Department of Surgical Oncology, Hospital Angeles, 5 Poniente 715, Puebla, Mexico; 3 Department of Radiology, Hospital Angeles, Puebla, México; 4 Department of Pathology, Valencia University, Valencia, Spain; 5 Current affiliation: Memorial Sloan-Kettering Cancer Center, New York, NY, USA

**Keywords:** Pulmonary artery, Sarcoma, Angiosarcoma, Immunohistochemistry

## Abstract

**Abstract:**

Primary sarcomas of the major blood vessels can be classified based on location in relationship to the wall or by histologic type. Angiosarcomas are malignant neoplasms that arise from the endothelial lining of the blood vessels; those arising in the intimal compartment of pulmonary artery are rare. We report a case of pulmonary artery angiosarcoma in a 36-year old female with pulmonary masses. The patient had no other primary malignant neoplasm, thus excluding a metastatic lesion. Gross examination revealed a thickened right pulmonary artery and a necrotic and hemorrhagic tumor, filling and occluding the vascular lumen. The mass extended distally, within the pulmonary vasculature of the right lung. Microscopically, an intravascular undifferentiated tumor was identified. The tumor cells showed expression for vascular markers VEGFR, VEGFR3, PDGFRa, FGF, Ulex europaeus, FVIII, FLI-1, CD31 and CD34; p53 was overexpressed and Ki67 proliferative rate was increased. Intravascular angiosarcomas are aggressive neoplasms, often associated with poor outcome.

**Virtual slide:**

The virtual slide(s) for this article can be found here: http://www.diagnosticpathology.diagnomx.eu/vs/2315906377648045.

## Background

Primary sarcomas of the major blood vessels can be classified based on location in relationship to the wall (mural or intraluminal (also known as “intimal”) or by histologic type. Angiosarcomas are malignant tumors that arise from the endothelial lining of the blood vessels [1]. Pulmonary artery sarcomas (PAS) include two types: intimal sarcomas, presenting as intraluminal growing excrescences, and mural sarcomas, involving the pulmonary artery wall. PAS are rare tumors, with unknown and probably, underestimated incidence, which may show myofibroblastic, leiomyosarcomatous, osteosarcomatous, rhabdomyosarcomatous or angiosarcomatous differentiation [2]. Angiosarcoma of the pulmonary artery is a distinctive tumor and few cases have been reported to the date [2,3].

The article "Pulmonary artery sarcoma with angiosarcoma phenotype mimicking pleomorphic malignant fibrous histiocytoma: a case report" was published in 2012. Journal: Diagn Pathol.

## Case presentation

A 36-year-old female presented to the clinic with a 3-month history of non-productive cough and weight loss. Her past medical history was unremarkable. Chest X-rays and a computed tomography (CT) scan showed two right perihilar lung masses, each measuring 3.5 and 2.5 cm in greater diameter, adjacent to the main right pulmonary artery (Figure 1). No extrapulmonary masses were identified by PET scan and CT; therefore, metastatic disease was excluded. A bronchoscopy was performed and transbronchial biopsies were taken but were non diagnostic. She had a thoracoscopic exploration and an open-lung biopsy. A pathology report showed a malignant fibrous histiocytoma (MFH) of the lung. A right pneumonectomy was performed and she required 2 days in the ICU; pulmonary artery hypertension and tachycardia developed, which resolved with digoxin and diltiazem.

**Figure 1:** **Pulmonary artery angiosarcoma. A** and **B**. CT-chest shows two circumscribed pulmonary masses.

### Pathological findings

The specimen consisted of a total right lung, weighing 994 grams and measuring 35 × 11 × 7 cm. On the anterior aspect of the right upper lobe, two masses that abut pleural surfaces were identified. Cut sections showed a right pulmonary artery thickening and a necrotic and hemorrhagic tumor, filling and near occluding the vascular lumen (Figure 2). The mass extended distally, within the pulmonary vasculature of the right lung. The smaller arterial branches were thickened. In addition, the lung parenchyma showed two lobulated and circumscribed yellow-tan masses with necrosis, hemorrhage and myxoid appearance, measuring 3.5 × 3.2 × 3 cm and 2.5 × 2 × 2 cm. The bronchial and vascular margins of resection were free of tumor.

**Figure 2:** **Pulmonary artery angiosarcoma. A**. Tumor abutting the pleural surface. **B**. Right pneumonectomy showing intraparenchymal masses and near total right pulmonary occlusion.

Microscopic examination showed an intravascular undifferentiated tumor composed of loosely cohesive large, pleomorphic spindle and epithelioid cells with prominent nucleoli, admixed with multinucleated giant cells (Figure 3). Numerous mitotic figures were seen. Interestingly, the pleomorphic tumor cells were found arising from the intima of the vessels, extending and occupying the vascular lumen. Medium sized vessels showed intraluminal tumor. Masson’s trichrome was useful to identify vessels components and the origin of tumor cells (not shown). The lung parenchyma also revealed a tumor similar that presented in pulmonary vessel, with solid, myxoid and hemangiopericytoid growth patterns. The original biopsy slides were reviewed, and the findings were identical to those identified within the vascular spaces and lung parenchyma. The original biopsy diagnosis was MFH pleomorphic variant.

The article "Pulmonary artery sarcoma with angiosarcoma phenotype mimicking pleomorphic malignant fibrous histiocytoma: a case report" was published in 2012. Journal: Diagn Pathol.

**Figure 3:** **Pulmonary artery angiosarcoma. A**, **B**. Endovascular tumor with intimal component (HE 40X, 10X). **C**, **D**. Intravascular angioblastic proliferation (HE 200X, 400X). **E**. Malignant tumor cells with vacuoles (HE 400X). **F**. Large epithelioid malignant tumor cells (HE 400X). **G**. Angioblasts within malignant vascular neoformation (HE 200X). **H**. Atypical endothelial proliferation (HE 400X).

A broad panel of immunohistochemical markers was used as shown in Table 1. The tumor cells showed strong positivity for Vimentin, FGF, PDGFRa, Factor VIII, Ulex europaeus, FLI1, CD31 and CD34; VE-cadherin, VEFGR and VEGFR3 were focal positive in epithelioid tumor cells; there was p53 overexpression (25%) and Ki67 proliferative rate ranged from 10 to 40% (Figure 4). Tumor cells lacked expression for AE1AE3, EMA, CK 8/18, HMB45, Melan A, desmin, h-Caldesmon, SMA and S100.

**Table 1:** List of antibodies

**ANTIBODY**	**CLONE**	**SOURCE**	**DILUTION**
VIMENTIN	Monoclonal mouse V9	Novocastra	1:300
CD31	Monoclonal mouse anti-h JC70A	DAKO	1:100
CD34	Monoclonal mouse QBEnd/10	Novocastra	1:100
VE-CADHERIN	Goat polyclonal	Santa cruz Biotechnology	1:100
VEGF	Mouse monoclonal VG1	Neomarkers	1:100
VEGFR3	Rabbit polyclonal	Santa cruz Biotechnology	1:400
PDGFRa	Rabbit polyclonal	Santa cruz Biotechnology	1:100
FGF-2	Rabbit polyclonal	Santa cruz Biotechnology	1:200
Factor VIII	Rabbit polyclonal	DAKO	1:200
ULEX EUROPAEUS-I LECTIN	Rabbit polyclonal	Sigma	1:500
FLI-1	Monoclonal mouse MRQ1	Cell Marque	1:100
EMA	Monoclonal mouse E29	DAKO	1:100
CK 8/18	Monoclonal mouse 5D3	Novocastra	1:50
CK AE1-AE3	Monoclonal mouse AE1-AE3	DAKO	1:100
S100	Rabbit polyclonal	DAKO	1:600
HMB45	HMB45	DAKO	1:100
Melan A	A103	DAKO	1:50
Desmin	DE-R11	DAKO	1:100
h-Caldesmon	Monoclonal mouse h-CD	DAKO	1:50
Ki67	Monoclonal mouse MIB-1	DAKO	1:200
P53	Monoclonal mouse DO-7	Novocastra	1:50

VE indicates vascular endothelial; VEGF, vascular endothelial growth factor; PDGFRa, platelet-derived growth factor receptor alpha; FGF, fibroblast growth factor; EMA, epithelial membrane antigen; CK, cytokeratin.

**Figure 4:** **Pulmonary artery angiosarcoma. A**. CD31 expression in tumor cells. **B**. CD34 highlights tumor cells. **C**. Strong positivity for Factor VIII. **D**. FLI-1 shows nuclear expression. **E**. Ulex europaeus positive staining. **F**. FGF expression. **G**. Ki67 nuclear staining. **H**. p53 nuclear staining.

Based on clinical, radiological and histopathological findings, the tumor was diagnosed as angiosarcoma arising on the pulmonary artery.

The article "Pulmonary artery sarcoma with angiosarcoma phenotype mimicking pleomorphic malignant fibrous histiocytoma: a case report" was published in 2012. Journal: Diagn Pathol.

### Clinical follow-up

The patient received four cycles of ifosfamide-based chemotherapy with tolerable toxicity. Eighteen months after diagnosis an extensive radiological examination showed no other primary neoplasm or metastatic lesion. The patient was disease free 18 months and then the tumor recurred (additional biopsies were taken showing similar histopathological findings). She developed metastatic disease to liver and contralateral lung and died 29 months after the recurrence. No autopsy was performed.

Primary sarcomas arising from major blood vessels (aorta, pulmonary artery, inferior vena cava) are exceedingly rare [4-8], and some of the cases presented in the literature have been autopsy reports [5,9,10]. Most patients are adults, however, a few cases have been found in children [11]. Burke *et al.*[5] found that intimal sarcomas affect males more frequently than females and arise predominatly in the right pulmonary vessels, with intraluminal involvement rather than intraparenchymal infiltration.

Clinically, primary sarcomas of the major blood vessels, are usually associated to embolic phenomena [6,12,13]; therefore, their true incidence is probably underestimated because of misdiagnosis with thromboembolism, especially when located at aorta [11]. The radiographic distinction of pulmonary thromboembolic disease and pulmonary artery sarcoma (PAS) is challenging, because both conditions appear as intraluminal filling defects in the pulmonary artery system on contrast-enhanced CT scans [14,15]. Some authors have reported that the diagnosis may be suspected by magnetic resonance imaging (MRI) [4,6] and positron emission tomography (PET) [15]. However, findings that favor a diagnosis of a PAS include the heterogeneous soft tissue density and the enhancement of the gadolinium contrast [11,16]. Therefore, PAS should always be considered as a possibility, as a misdiagnosis with thromboembolic disease will result in delaying appropriate therapy and increased morbi-mortality [15,17].

Grossly, a careful examination of the specimen, the pulmonary vasculature and its branches is essential to achieve the correct diagnosis. PAS may spread and grow as intraluminal masses along the endothelium and an organizing thromboemboli needs to be ruled out [18]. In addition, direct lung parenchyma involvement is a common event, as direct extension through the pulmonary vasculature can occur due to the prominent intravascular growth along the arterial intima. On the other hand, mural sarcomas with a solid growth can also be confused with other entities including metastatic extension from primary malignancies of the lung or tumors from the mediastinum, such as lymphoma and sarcomas [19]. In our case, an extensive work-up that included clinical and radiological evaluation was a key determinant for the appropriate conclusion of the case.

The article "Pulmonary artery sarcoma with angiosarcoma phenotype mimicking pleomorphic malignant fibrous histiocytoma: a case report" was published in 2012. Journal: Diagn Pathol.

Pulmonary artery sarcomas of the lung are malignant tumors of indeterminate cause, usually presenting heterogenous histology that most likely reflect a pluripotential or mesenchymal cell origin [20]. Some examples that have been reviewed in the literature represent undifferentiated sarcomas that may display a myofibroblastic or leiomyosarcomatous component [5,18]; nevertheless, osteosarcomatous, chondrosarcomatous, rhabdomyosarcomatous, liposarcomatous and angiosarcomatous elements have also been described [5,6,8-10,21-23]. The present case displays an undifferentiated sarcoma that mimics pleomorphic malignant fibrous histiocytoma; however, the tumor expresses the majority of vascular-specific markers. It is important to highlight that the final diagnosis could not have been achieved without a high level of suspicion. Interestingly, one of the most significant features helpful for identification of angiosarcoma was the intimal origin of the tumor. Furthermore, undifferentiated tumors as primary pulmonary angiosarcomas have been confused with malignant neoplasms (primary or metastatic malignancies) with dedifferentiated component, such as carcinomas, sarcomas and lymphomas [24-27]. Differential diagnoses in this specific case include high grade sarcomas with leiomyosarcomatous, fibro or myofibroblastic differentiation. For that reason, an appropriate and consecutive utilization of a broad panel of antibodies, and occasionally, electron microscopy (not used in this case) are often necessary to distinguish the origin [8,13,28]. We found in this case, that co-expression of endothelial markers such as VEGF, PDGFR, Ulex europaeus, FLI1, CD31 and CD34 is useful in classifying the neoplasm, representing an unusual presentation of a true angiosarcoma similar to those observed in soft tissues.

Although in this case it was not possible to identify specific exposure, angiosarcomas have been reported associated to previous irradiation fields [29] or arteriovenous fistulas [30]. Comparative genomic hybridization (CGH) analysis of intimal pulmonary sarcomas have shown gains and amplifications in the 12q13–14 region, with other less consistent findings including losses on 3p, 3q, 4q, 9p, 11q, 13q, Xp, and Xq, gains on 7p, 17p, and 17q, and amplifications on 4q, 5p, 6p, and 11q [18]. Currently, no prognostic markers have been extensively studied; however, in one study, Gaumann *et al.*[31] found that osteopontin expression may contribute to metastasis due to its role in cell attachment and therefore to poor prognosis. In addition, Bode-Lesniewska *et al.*[18] reported that dysregulation of the cell cycle proteins in p53 pathway and overexpression of mdm2 might be implicated in the pathogenesis. At this point, further gene profiling studies, including a larger group of this specific type of vascular malignancy can be used to identify predictive and prognostic markers for intravascular angiosarcoma of the pulmonary vessels.

The article "Pulmonary artery sarcoma with angiosarcoma phenotype mimicking pleomorphic malignant fibrous histiocytoma: a case report" was published in 2012. Journal: Diagn Pathol.

Overall, PAS are considered aggressive neoplasms, often associated to poor outcome irrespective of treatment [9,10,32,33], and with no exception for pulmonary artery angiosarcomas. Only few patients have survived more than 12 months [5,34]; surgery and complete resection of the tumor provide local control. Adjuvant chemotherapy and radiotherapy have a controversial role in the management of this disease [5,33]. The role of chemotherapy is unclear, but a 50% response rate has been found to palliative chemotherapy with anthracyclines and ifosfamide in patients with advanced PAS [11,35].

## Conclusion

In summary, we report an unusual case of pulmonary artery sarcoma with angiosarcoma phenotype that mimics pleomorphic malignant fibrous histiocytoma. A high level of suspicion and identification of the intimal location of the tumor, in addition to the use of a broad panel of immunohistochemical markers were helpful for the identification of the vascular origin. A multidisciplinary clinical and radiological approach and an extensive work-up were key determinant for the appropriate conclusion of the case.

## Consent

Written informed consent was obtained from the patient’s family members for publication of this Case Report and any accompanying images. A copy of the written consent is available for review by the Editor-in Chief of this journal.

## Competing interests

The authors declare that they have no competing interests.

## Authors’ contributions

OB, EA, OL, NR, SS and AL have been directly involved in diagnosis and interpretation of patient’s diagnosis. OB, SS and AL were responsible for the conception and design of the Case Report. All authors read and approved the final manuscript.
